# Antidepressant Mechanism of Kaixinsan and Its Active Compounds Based on Upregulation of Antioxidant Thioredoxin

**DOI:** 10.1155/2022/7302442

**Published:** 2022-07-19

**Authors:** Xia Li, Yuan-bo Wang, Chao-chen Wang, Rui Jing, Li-hua Mu, Ping Liu, Yuan Hu

**Affiliations:** ^1^Department of Pharmacy, Medical Supplier Center of PLA General Hospital, Beijing 100853, China; ^2^Graduate School of PLA General Hospital, Beijing 100853, China

## Abstract

**Objectives:**

Kaixinsan (KXS), a traditional Chinese medicine formula, has been demonstrated to be effective in the treatment of depression. The present study applied a network pharmacology approach to dig out the new targets and mechanism of action of KXS and the active compounds in the treatment of depression.

**Methods:**

A network pharmacology approach based on public databases including ADME (absorption, distribution, metabolism, and excretion) evaluation, targets prediction, construction of networks, and molecule docking was used and validated the predicted new antioxidant targets and mechanisms in vitro. Based on an in vitro experiment, we verified the AKT1/Nrf2 pathway related to the thioredoxin (Trx) antioxidant mechanism.

**Results:**

The present study sorted 31 pharmacologically active components (kaempferol, ginsenoside rh2, ginsenoside rh4, stigmasterol, etc.) through the ADME algorithm from KXS. 136 potential molecular targets (AKT1, TNF, IL-1b, JUN, ESR1, NOS3, etc.) were predicted, of which there were 69 targets clearly related to depression. By compound-depression targets (C-DTs) network constructed, and protein-protein interaction networks (PPI) and KEGG pathway enrichment analyzed, we identified active compounds mediating depression-related targets to exert synergism on the predictive AKT1/Nrf2 pathway related to thioredoxin (Trx) antioxidant mechanism and other inflammation-related signaling pathways as well as neurotransmitter related signaling pathways. In the H_2_O_2_ induced SH-SY5Y cell damage model, this showed kaempferol and ginsenoside rh2 could enhance the activity of the Trx system by upregulation of AKT1 to activate Nrf2 in vitro.

**Conclusions:**

Taken together, by comprehensive systems pharmacology approach analysis, we found that KXS and its active compounds might exhibit antioxidant effects by stimulating the AKT1/Nrf2 pathway in the treatment of depression, which might shed new light on innovative therapeutic tactics for the new aspects for depression in traditional Chinese medicine in future studies.

## 1. Introduction

Depression has huge social risks of high incidence, disability, and suicide. At present, the main clinical antidepressants are selective 5-HT reuptake inhibitors, tricyclic or tetracyclic antidepressants, and monoamine oxidase inhibitors. Chronic treatment with antidepressants is only 60 to 70 percent effective with significant side effects [1].

With a long history of thousands of years, traditional Chinese medicine (TCM) plays important roles in the treatment of mental illness. Natural products, such as plants, animals, and minerals, are typically prescribed in TCM, in which herbal or botanical products are most widely used. Depression can be traced back to the traditional Chinese medicine book “Huang Di Nei Jing” more than 2000 years ago, which belongs to the category of “depressive syndrome-YuZheng” in TCM. TCM shows its advantage for containing a variety of chemical components, which targets through various channels, and significantly alleviating complications such as insomnia and anxiety while treating depression.

In fact, the serotonergic, dopaminergic, and noradrenergic systems are deeply involved in the mechanisms of TCMs' antidepression process. Among them, inhibition against monoamine oxidase reaction and increasing synaptic availability of monoamines are the main factors in TCMs' monoamine regulation mechanism. For example, Xiaoyaosan could improve the serotonergic metabolism by regulating the expression levels of tryptophan hydrogenase 2 (TPH2) and indoleamine 2,3-dioxygenase 1 (IDO1), thus exerting an antidepressant effect [2]. The antidepressant-like effect was also the main function in the Banxia-Houpu decoction by attenuating abnormalities in the serotonergic and dopaminergic system functions in animal models of depression [3]. The antidepressant effect of Kaixinsan (KXS) could be explained by modulation of the noradrenergic system and the 5-hydroxytryptamine (5-HT) system in mice as well [4]. Other than the neurotransmitter mechanism, depression is triggered by other complicated pathogenetic factors such as oxidative stress. Chronic SNRI\SSRI treatment in effective antidepressant doses was shown to protect against chronic stress-increased oxidative cellular or DNA damage and inhibited reactive oxygen species (ROS) and lipid peroxidation levels in the hippocampus [5], and this mechanism might rely on the AKT /Nrf2/HO-1 pathway [6]. These results indicated that inhibition of oxidative stress played a vital role in the pathogenesis of depression. Therefore, there might be a novel way to evaluate the therapeutic effects and mechanisms of TCM and its active compounds.

KXS is a classic ancient prescription, first recorded the “Qianjin Yaofang” written by Sun Simiao in the Tang Dynasty. It is composed of *Ginseng Radix* (*Panax ginseng C. A. Mey.*), *Polygalae Radix* (*Polygala tenuifolia Wild.*), *Poria* (*Poria cocos (Schw.) Wolf*), and *Acori Tatarinowii Rhizoma* (*Acorus tatarinowii Schott*), with different ratio. As our previous clinical trials showed that KXS (3 : 3 : 2 : 2 ratios) ameliorated clinical symptoms of patients with minor and modest depression [7]. Pharmacological studies indicated that KXS significantly reduced depressive-like behavior on the forced swim test, the open-field test, in the CUMS animal models. It mainly focused on the mechanism of neurotransmitter regulation, or alleviating the hypothalamic-pituitary-adrenal (HPA) axis dysfunctions, lightening the impairment of neuroplasticity, and inflammatory regulation [8]. Although some studies have confirmed that some of the active compounds from the formula plants like ginsenoside rg1, ginsenoside rk1, polygalaxanthone III, essential oil, and polysaccharides from *Ginseng Radix* [9, 10], *Polygalae Radix* [11], *Acori Tatarinowii Rhizoma* [12] and *Poria* [13] have an obvious antioxidant effect. However, the rather complicated multicomponent compounds of KXS and its antioxidant molecular mechanisms are yet to be revealed.

Herein, we screened the potential active compounds of the four herbs contained in KXS with the computational ADME and selected depression-related targets, then combined the KEGG enrichment analysis and PPI were performed illustrate its possible mechanisms, especially those involved with oxidant stress, and finally performed to reveal the potential compounds in KXS on its specific antioxidant pathway. The work scheme of this research is shown in Figure 1.

## 2. Materials and Methods

### 2.1. Acquisition of the Active Compounds and Prediction of the Targets

According to the database TCMSP (https://tcmspw.com/tcmsp.php) [14], TCMID (http://119.3.41.228:8000/tcmid/search/) [15], and Symmap (https://www.symmap.org/) [16], the effective compounds of the four herbs *Ginseng Radix*, *Polygalae Radix*, *Poria*, and *Acori Tatarinowii Rhizoma* contained in KXS were screened. According to the ADME algorithm, oral bioavailability (OB) ≥30% and drug-likeness (DL) ≥0.18 were set as the screening criteria, and the active compounds, MolID, and action targets of the herbs were finally obtained. The same repeated active compounds and their action targets in the four herbs were combined using Venny 2.1.0 (https://bioinfogp.cnb.csic.es/tools/venny/) online software to obtain the effective compounds and targets in the KXS.

### 2.2. Protein-Protein Interaction Networks of Common Targets between KXS and Depression

The Disgenet (https://www.disgenet.org) [17] database selected the depression-related targets. The depression search terms were “mental depression” and “depression.” The same targets of depression were obtained after KXS treatment with Venny 2.1.0 online software. The Uniprot (https://www.uniprot.org/) [18] database converted KXS targets related to depression into international common gene names, and Uniprot IDs were obtained. Using String 11.0 (https://string-db.org/), the obtained common targets of KXS in the treatment of depression were visualized, and the protein-protein interaction networks (PPI) were drawn.

### 2.3. KEGG Pathway Analysis

The KEGG database (https://www.kegg.jp/) [19] conducted a KEGG pathway analysis on the common targets of KXS in the treatment of depression. *P* < 0.05 was set, the species was limited to homo sapiens, the top 10 targets related to KEGG pathway enrichment were listed, and the antioxidant pathways were found.

### 2.4. Molecular Docking

The Autodock Vina software calculated the free energy of molecular docking between the selected key targets and the corresponding compounds of KXS. The Pymol software was used for mapping, and the results of molecular docking were visualized to verify the network pharmacological analysis.

### 2.5. Cell Culture and Drug Treatment

The human neuroblastoma SH-SY5Y cells were selected to construct the model of oxidant stress damage in vitro. The cell-complete medium was DMEM supplemented with 10% fetal bovine serum. SH-SY5Y cell suspension with a concentration of 5 × 10^5^/mL and a volume of 100 *μ*L in the logarithmic growth phase was added to the 96-well plate. After screening the H_2_O_2_ induced damage concentration, it is set on 100 *μ*mol/L to induced injury model. Then, the active compounds kaempferol and ginsenoside rh2 with different dosages were added to the cell for 24 h. Four groups were set up: untreated control group, H_2_O_2_ induced injury model group, kaempferol treatment group, and ginsenoside rh2 treatment group.

### 2.6. Cell Viability

The cell viability was measured with the Cell Counting Kit-8 (CCK8) Assay (Beyotime). The SH-SY5Y cells (1 × 10^5^) were cultured in an incubator with 5% CO_2_ at 37°C for 24 h under different treatments in the 96-well plate. Totally 10 *μ*L CCK8 solution was added into each well, and the cells were cultured for another 1 h. The absorbance was finally determined at 450 nm with a microplate reader.

### 2.7. Western Blot

The SH-SY5Y cells were inoculated in the six-well plate after four ways of treatment, and 100 *μ*L RIPA lysis buffer was inoculated in each well. The cells were blown evenly and shaken evenly in a 4°C shaker for 30 min. Then the cells were scraped with a scraper and divided into EP tubes. The protein concentration was detected by the BCA method on each sample. After 1.5 *μ*g/*μ*L loading of the samples, they went to SDS-PAGE gel electrophoresis, transferred to PVDF membrane, and closed. After elution, the primary antibody AKT1 (diluted 1 : 1500, Beyotime, catalog no.AF1777), Nrf2 (diluted 1 : 1000, Beyotime, catalog no.AF7623), Trx (diluted 1 : 500, Servicebio, catalog no.GB11957) were incubated overnight, and then incubated the (HRP)-conjugated secondary antibody (diluted 1 : 1000, Beyotime, catalog no.A0208). Immunoblots were visualized by BeyoECL Plus kit (Beyotime, catalog no.P0018S) and quantified by densitometry in the western blotting detection system (UVP EC3 chemi HR 410 imaging system, California USA) and ImageJ software (National Institutes of Health).

### 2.8. Activity of Thioredoxin Reductase (TrxR) Determination

The activity of TrxR was measured by the Solarbio thioredoxin reductase activity Kit. We used 2-vinylpyridine to inhibit the original reduced glutathione in each sample. The activity of TrxR was calculated by measuring the absorbance at 412 nm.

### 2.9. Statistical Analysis

Statistical data were analyzed by GraphPad Prism 5 and compared with a one-way analysis of variance. The bilateral 95% confidence interval was used for all tests, and a value of *P* < 0.05 represented statistical significance.

## 3. Results

### 3.1. Active Compounds and Targets of KXS Screening

17 effective compounds of *Ginseng Radix* were screened, and 117 targets were identified. 6 effective compounds of *Poria* were screened, and 25 targets were identified. 4 effective compounds of *Acori Tatarinowii Rhizoma* were screened, and 81 targets were identified. 5 effective compounds of *Polygalae Radix* were screened, and 31 targets were identified (Figure 2(c)). By using Venny 2.1.0 online software, After removing repetitive compounds and targets, we finally obtained 30 active compounds in KXS with 134 targets(Figures 2(a) and 2(b)). As a review of the literature, *Ginseng Radix*, *Polygalae Radix*, *Poria*, and *Acori Tatarinowii Rhizoma* belonged to adaptogenic plants, so that all of the compounds could be classified into three main chemical groups, with a tetracyclic skeleton-like cortisol and testosterone, structural analogs of catecholamines or tyrosine and structural analogs of resolvins according to the criteria [20] (Table 1).

### 3.2. Protein-Protein Interaction Networks of Compound-Depression Targets (C-DTs)

Disgenet database screened depression targets and 1479 depression-related targets were obtained. According to the Venn diagram, there were 69 related targets of depression and KXS (Figure 3(a)). According to STRING 11.0 protein interactions, the network of 69 targets related to the treatment of depression by KXS was extensively connected with AKT1 as the core. A node represents one protein, and the degree value determines the size of the node. PPI also proved that AKT1 was much more likely to be a key target in this network. Among the targets, there were antioxidant-related targets, such as AKT1 (RACalpha serine/threonine-protein kinase, degree = 43), NOS3 (Nitric-oxide synthase, endothelial, degree = 28), Nrf2 (Nuclear factor erythroid 2-related factor 2, degree = 18)) and KEAP1 (Kelch-like ECH-associated protein 1, degree = 18) with a high degree, which initially proved that antioxidant active the important role in KXS antidepressive treatment (Figure 3(b)).

### 3.3. Functional and Pathway Enrichment Analysis and Antioxidant Pathway Identification

The KEGG pathway analysis of the related targets of KXS in the treatment of depression was performed by the KEGG database, and the tissue origin was limited to homo sapiens. The result showed that target genes were mapped into 227 pathways. The top 10 significantly enriched (adjusted *P* < 0.05) signaling pathways were preserved for further analysis. Multiple signaling pathways were involved in the treatment of depression with KXS, including pathways in cancer and metabolic pathways, and neurotransmitter-related pathways (Figure 4(a)). Based on the results of pathway analysis, besides the first two high-degree pathways, which were related to caner and the prime central nervous system function, it was found that the third pathway was closely related to the fluid shear stress and atherosclerosis pathway which included AKT1/Nrf2 pathways. Further analysis found that AKT1/Nrf2 pathways play an important role in antioxidant function, which could achieve antioxidant effects by influencing the activation of Thioredoxin (Trx) (Figure 4(b)).

### 3.4. Molecular Docking Validation of Selected Compound-Target Interactions

The molecular docking free energy of a ligand was associated with the number and strength of its binding forces with its receptor. Through molecular docking analysis, antioxidant targets as probes for validation of the compound-Target interactions of the formula were screened. At last, we used ligands and binding sites for molecular docking to verify whether the compound and target have good binding activity. The results showed that ginsenoside rh2 and AKT1, kaempferol, and AKT1 had larger free energy (Table 2). The molecular docking images of ginsenoside rh2 and AKT1, kaempferol, and AKT1 showed a high degree of fitting (Figure 5). According to the results, we speculated that AKT1 might be the key target of kaempferol and ginsenoside rh2, which is also the hub core gene in the PPI network. Therefore, we predicted kaempferol and ginsenoside rh2 as potential active compounds of KXS involved in its antioxidant mechanism.

### 3.5. Experimental Validation of Active Compounds in KXS Protected Oxidative Stress Induced Damage in SY5Y Cells by Increased the Antioxidant TrxR Activity

In Figure 6, both kaempferol and ginsenoside rh2 significantly inhibited 100 *μ*mol/L H_2_O_2_ induced SY5Y cell damage, at 25 *μ*mol/L and 40 *μ*mol/L, respectively. At the same time, H_2_O_2_ (100 *μ*mol/L) in 24 h induced a significant increase of TrxR activity, compared with the control group, and then decreased at 72 h, which might be a process of depletion. Kaempferol and ginsenoside rh2 kept the activity of TrxR from 24 h to 72 h, compared with H_2_O_2_ induced damage group, indicating they might keep the Trx protein system maintained for stronger antioxidant capacity for a longer time. And the antioxidant effect of kaempferol was significantly better than that of ginsenoside rh2.

### 3.6. Keampferol and Ginsenoside rh2 Exerted Antioxidant Functions Through AKT1/Nrf2 Pathwaysz

According to the retrieval of Trx protein-related pathways in the KEGG database, AKT1 and Nrf2 were the upstream proteins in the antioxidant pathway of Trx. Here, the results indicated that kaempferol and ginsenoside rh2 could increase the expression of Trx protein. Meanwhile, these two monomer compounds could also increase the expression of AKT1 and Nrf2, which boosted the targets in the AKT1/Nrf2/Trx pathways cascade working together. Similar to Trx activity, kaempferol works better than that of ginsenoside rh2 in the AKT1 /Nrf2/Trx pathways (Figure 7).

## 4. Discussion

According to our results, by systems pharmacology approach which contained ADME screening, targets prediction, network analysis, and pathway screening, we verified the “multicompound, multitarget, and multipathway” properties of the KXS formula. We identified depression-associated targets of KXS compounds, among them AKT1 was identified as core antidepressive target of KXS. More specifically with its antioxidant mechanism, we found that KXS and its anti-oxidant monomer compounds might work on AKT1/Nrf2 pathways to activate the Trx antioxidant system. According to the results, the advantages of KXS for treating depression mainly concentrate on the following aspects.

Firstly, the active compounds of the KXS formula are large in number, which might greatly increase the multitarget effect and reduce the possibility of side effects and drug resistance. KXS takes flavonoids, saponins, oligosaccharides, polysaccharides, and volatile oil as the main active compounds [21], and its antidepressant pharmacology and compound studies have made certain progress [22, 23]. By network pharmacology analysis, kaempferol and ginsenoside rh2 were recognized as key compounds of KXS. Ginsenoside rh2 belongs to compounds with a tetracyclic skeleton and kaempferol belongs to structural analogs of catecholamines. Kaempferol is a kind of flavonoid, which can inhibit oxidative stress and cell apoptosis. It has been shown to have protective effects on depression models. It exerts antidepressive effects, which might be mediated by enhanced antioxidant abilities and anti-inflammation effects in the prefrontal cortex of CSDS mice [24]. Ginsenoside rh2 is a secondary ginsenoside produced by the decomposition of some proto-ginsenosides by heat, resulting in the degradation of the sugar chain on their ligands. It was confirmed that ginsenoside rh2 can significantly down-regulate the levels of TNF-*α* and IL-6 in the serum of depressed mice, and up-regulate the activity of superoxide dismutase (SOD) in the hippocampus [25]. These references suggest the potential of these two compounds in antioxidant studies.

Secondly, many studies had shown that the mechanism of KXS in the treatment of depression was to improve the activity of neurotransmitters such as 5-HT [26] and acetylcholine [27], repair the secretion decline of neurotrophic factors such as BDNF [28] and NGF [29] or their related signaling pathway damage, reduce the level of central nervous inflammatory factors such as inhibiting the increase of IL-1*β*, IL-6, and TNF-*α* [30], and increase the activity of superoxide dismutase to reduce lipid peroxidation, protecting hippocampal nerve cells. Further review of the literature showed that KXS, as a traditional Chinese medicine prescription for the treatment of emotional diseases, was also effective in the treatment of Alzheimer's disease(AD) in addition to depression. KXS could reduce the deposition of amyloid *β*-protein (A*β*) [31], improve the plasticity of neurons [32], inhibit the activity of acetylcholinesterase, and significantly improve mitochondrial function by reducing ROS levels and increasing mitochondrial membrane potential [33]. These studies suggest that the antioxidant mechanism of KXS plays an important role in the treatment of emotional diseases, including depression. However, most studies on the antioxidant mechanism are relatively superficial and lack of in-depth explanation. So, we mainly explored the antioxidation-related mechanisms by KEGG pathway enrichment analysis. We found that antioxidant-related targets AKT1, NOS3, Nrf2, and KEAP1 have high research potential and KXS could activate the AKT/Nrf2 pathway to up-regulate the activity of several antioxidant systems, such as glutathione (GSH) system [34], reactive oxygen species (ROS) [35], heme oxygenase(HO) system [36], and Trx system. These antioxidant mechanisms may play an important role in the treatment of depression.

Thirdly, most studies on the antioxidation of antidepressants focused on the GSH system, ROS, and HO systems. The mechanism of antioxidants was mainly on Trx antioxidant system, relatively less studied. The Trx system is a small molecule protein system associated with redox action in the body. This system is composed of Trx, thioredoxin reductase (TrxR), and nicotinamide adenine dinucleotide phosphate (NADPH). It can reduce the cysteine residues of oxidized Trx and further acts as an electron donor for ribonucleotide reduction, maintaining its antioxidant capacity [37], so that it is an important participant in antioxidant free radicals, antiapoptosis, and promoting cell growth in cells. Several reports have shown that Trx has an obvious antioxidant effect [38, 39], and the serum content of Trx is decreased in patients with depression. As the preclinical systematic review study found, KXS, most treated for Alzheimer's Disease and Depression, has an effect on antioxidant activity by decreased ROS and MDA levels via increased GSH and SOD levels. Here, in a combined analysis of the KXS antidepressive related targets identifying and targets pathway, we illustrated the potential AKT/Nrf2/Trx pathway as a novel antioxidant mechanism of KXS therapy. Furthermore, found that kaempferol and ginsenoside rh2 as effective compounds of KXS protected H_2_O_2_ oxidative damage of SH-SY5Y cells in vitro, and instantly keeping enhanced the activity of Trx by increasing its upstream proteins AKT1 and Nrf2. While, the antioxidant effect of kaempferol is better than that of ginsenoside rh2, which makes kaempferol become a valuable active compound with new targets for treating depression. Of course, there are some deficiencies in this study. For example, the components and effective targets of KXS after screening by ADME are relatively few, and only in vitro model studies have been carried out. There is still a lot of work to be made up in the following studies.

In conclusion, for the first time, we identified the AKT/Nrf2 pathway and targets of KXS compounds using an integrative systems pharmacology approach. Furthermore, we validated the mechanisms by which KXS and its active compound ameliorated depression as shown in Figure 8.

## Figures and Tables

**Figure 1:** The flowchart of the entire research procedure.

**Figure 2:** Diagram of active compounds in KXS: (a) targets of the four herbs in KXS. (b) Effective compounds of the four herbs in KXS. (c) compounds to target the interaction diagram of the four herbs. In the figure, the red icons represent the herbs, the yellow icons represent the compounds, and the green icons represent the targets. The larger the icons area is, the greater the degrees in the interaction network are, indicating that the targets play a more important role in the network).

**Figure 3:** Diagram of KXS targets in the treatment of depression: (a) Venn diagram of KXS targets in the treatment of depression; (b) protein-protein interaction networks).

**Figure 4:** KEGG pathway analysis, (a) In the first 10 KEGG pathways, analysis of KXS in the treatment of depression, the size of each node indicates enriched counts. Abscissa represents the enriched gene count. Color means enriched adjust *P*-value. (b) Activation of AKT1/Nrf2 pathway network in the treatment of KXS).

**Figure 5:** Images of molecular docking. (a) Molecular docking of kaempferol and AKT1; (b) molecular docking of ginsenoside rh2 and AKT1; (c) molecular docking of 1,7-dihydroxy-3-methoxy xanthone and GSK3B; (d) molecular docking of 8-isopentenyl-kaempferol and ESR1; (e) molecular docking of trametenolic acid and NR3C2; (f) molecular docking of stigmasterol and NR3C2).

**Figure 6:** Kaempferol and ginsenoside rh2 increased the cell viability and the activity of antioxidant TrxR in vitro: (a) screening the best concentration of H_2_O_2_ in SY5Y cells; (b) the cell viability of kaempferol treatment with different doses; (c) the cell viability of ginsenoside rh2 treatment with different doses; (d) TrxR activity in SY5Y cells induced by H_2_O_2_ at different treatment time; (e) kaempferol and ginsenoside rh2 increased TrxR activity induced by H_2_O_2_ in 24 h; (f) kaempferol and ginsenoside rh2 increased TrxR activity induced by H_2_O_2_ in 72 h.^*∗*^*p* < 0.05 vs.H_2_O_2_ model group; ^*∗∗*^*p* < 0.01 vs.H_2_O_2_ model group; ^##^*p* < 0.01 vs. control group). Kaempferol and ginsenoside rh2 exerted antioxidant functions through AKT1 /Nrf2 pathways.

**Figure 7:** Kaempferol and ginsenoside rh2 up-regulated the expression of AKT1, Nrf2 and Trx proteins in vitro: (a) kaempferol and ginsenoside rh2 up-regulated AKT1 expression; (b) kaempferol and ginsenoside rh2 up-regulated Nrf2 expression; (c) kaempferol and ginsenoside rh2 up-regulated Trx expression. Data represented the means ± SEM, ^#^*P* < 0.05 vs. the control group; ^*∗*^*P* < 0.05, ^*∗∗*^*P* < 0.01 vs. the model group).

**Figure 8:** Pathway for kaempferol and ginsenoside rh2 to activate the Trx system.

**Table 1:** Summary of compounds in KXS (I: compounds with a tetracyclic skeleton-like cortisol and testosterone; II: structural analogs of catecholamines or tyrosine; III: structural analogs of resolvins).

Mol ID	Compound	Herb	OB (%)	DL	Chemical formula	Chemical group
MOL002879	Diop	*Ginseng Radix*	43.59	0.39	C_24_H_38_O_4_	III
MOL000449	Stigmasterol	*Ginseng Radix*	43.83	0.76	C_29_H_48_O	I
MOL000358	Beta-sitosterol	*Ginseng Radix*	36.91	0.75	C_29_H_50_O	I
MOL003648	Inermin	*Ginseng Radix*	65.83	0.54	C_16_H_12_O_5_	II
MOL000422	Kaempferol	*Ginseng Radix Acori Tatarinowii Rhizoma*	41.88	0.24	C_15_H_10_O_6_	II
MOL005308	Aposiopolamine	*Ginseng Radix*	66.65	0.22	C_17_H_19_NO_3_	II
MOL005317	Deoxyharringtonine	*Ginseng radix*	39.27	0.81	C_28_H_37_NO_8_	II
MOL005318	Dianthramine	*Ginseng radix*	40.45	0.20	C_14_H_11_NO_6_	II
MOL005320	Arachidonate	*Ginseng radix*	45.57	0.20	C_20_H_32_O_2_	III
MOL005321	Frutinone A	*Ginseng Radix、Polygalae Radix*	65.9	0.34	C_16_H_8_O_4_	II
MOL005344	Ginsenoside rh2	*Ginseng Radix*	36.32	0.56	C_36_H_62_O_8_	I
MOL005348	Ginsenoside-Rh4	*Ginseng Radix*	31.11	0.78	C_36_H_60_O_8_	I
MOL005356	Girinimbin	*Ginseng Radix*	61.22	0.31	C_18_H_17_NO	II
MOL005376	Panaxadiol	*Ginseng Radix*	33.09	0.79	C_30_H_52_O_3_	I
MOL005384	Suchilactone	*ginseng Radix*	57.52	0.56	C_21_H_20_O_6_	II
MOL005399	Alexandrin	*Ginseng Radix*	36.91	0.75	C_35_H_60_O_6_	I
MOL000787	Fumarine	*Ginseng Radix*	59.26	0.83	C_20_H_19_NO_5_	II
MOL000273	(2R)-2-[(3S 5R 10S 13R 14R 16R 17R)-3,16-Dihydroxy-4 4 10 13 14-pentamethyl-2 3 5 6 12 15 16 17-octahydro-1H-cyclopenta[a]phenanthren-17-yl]-6-methylhept-5-enoic acid	*Poria*	38.26	0.82	C_30_H_46_O_4_	I
MOL000275	Trametenolic acid	*Poria*	38.71	0.80	C_30_H_48_O_3_	I
MOL000279	Cerevisterol	*Poria*	37.96	0.77	C_28_H_46_O_3_	I
MOL000282	Ergosta-7 22E-dien-3beta-ol	*Poria*	43.51	0.72	C_28_H_46_O	I
MOL000283	Ergosterol peroxide	*Poria*	40.36	0.81	C_28_H_44_O_3_	I
MOL000296	Hederagenin	*Poria*	36.91	0.75	C_30_H_48_O_4_	I
MOL002140	Perlolyrine	*Polygalae Radix*	65.95	0.27	C_16_H_12_N_2_O_2_	II
MOL004718	*α*-Spinasterol	*Polygalae Radix*	42.98	0.76	C_29_H_48_O	I
MOL013171	1 6-Dihydroxy-3 7-dimethoxyxanthone	*Polygalae Radix*	89.65	0.27	C_15_H_12_O_6_	II
MOL003152	1 7-Dihydroxy-3-methoxy xanthone	*Polygalae Radix*	64.06	0.21	C_14_H_10_O_5_	II
MOL003542	8-Isopentenyl-kaempferol	*Acori Tatarinowii Rhizoma*	38.04	0.39	C_20_H_18_O_6_	II
MOL003576	(1R 3aS 4R 6aS)-1 4-bis (34-dimethoxyphenyl)-1 3 3a 4 6 6a-hexahydrofuro [4 3-c] furan	*Acori Tatarinowii Rhizoma*	52.35	0.62	C_22_H_26_O_6_	II
MOL003578	Cycloartenol	*Acori Tatarinowii Rhizoma*	38.69	0.78	C_30_H_50_O	I

**Table 2:** Molecular docking of KXS in the treatment of depression (the first 21 groups) (the molecular docking free energy is negative, which theoretically indicates that the drug compounds can bind to the target in the natural state, and the greater the absolute value of the negative value indicates the stronger the binding ability).

Compound	Herb	Target	Free energy
Kaempferol	*Ginseng Radix, Acori Tatarinowii Rhizoma*	AKT1	−9
Ginsenoside rh2	*Ginseng Radix*	AKT1	−8.2
1,7-Dihydroxy-3-methoxy xanthone	*Polygalae Radix*	GSK3B	−7.5
8-Isopentenyl-kaempferol	*Acori Tatarinowii Rhizoma*	ESR1	−7.4
Trametenolic acid	*Poria*	NR3C2	−7.1
Stigmasterol	*Ginseng Radix*	NR3C2	−6.9
Kaempferol	*Ginseng Radix, Acori Tatarinowii Rhizoma*	Nrf2	**−6.9**
Kaempferol	*Ginseng Radix, Acori Tatarinowii Rhizoma*	KEAP1	**−6.8**
Cerevisterol	*Poria*	NR3C2	−6.7
Beta-sitosterol	*Ginseng Radix*	BAX	−6.6
Kaempferol	*Ginseng Radix, Acori Tatarinowii Rhizoma*	BAX	−6.6
Kaempferol	*Ginseng Radix, Acori Tatarinowii Rhizoma*	NOS3	**−6.5**
Cycloartenol	*Acori Tatarinowii Rhizoma*	NR3C2	−6.2
*α*-Spinasterol	*Polygalae Radix*	NR3C2	−6.2
1,7-Dihydroxy-3-methoxy xanthone	*Polygalae Radix*	NOS2	−6
1,6-Dihydroxy-3,7-dimethoxyxanthone	*Polygalae Radix*	NOS2	−6
(2R)-2-[(3S,5R,10S,13R,14R,16R,17R)-3,16-dihydroxy-4,4,10,13,14-pentamethyl-2,3,5,6,12,15,16,17-octahydro-1H-cyclopenta[a]phenanthren-17-yl]-6-methylhept-5-enoic acid	*Poria*	NR3C2	−5.8
Deoxyharringtonine	*Ginseng Radix*	NR3C2	−5.8
Ginsenoside rh4	*Ginseng Radix*	NR3C2	−5.7
Ginsenoside rh2	*Ginseng Radix*	Nrf2	**−5.6**
Ginsenoside rh2	*Ginseng Radix*	KEAP1	**−5.3**

## Data Availability

This study is based on the public databases TCMSP (https://tcmspw.com/tcmsp.php), TCMID (http://119.3.41.228:8000/tcmid/search/), Disgenet (https://www.disgenet.org), Uniprot (https://www.uniprot.org/), KEGG (https://www.kegg.jp/), and Symmap (https://www.symmap. org/).

## References

[1] Oremus C., Oremus M., McNeely H. (2015). Effects of electroconvulsive therapy on cognitive functioning in patients with depression: protocol for a systematic review and meta-analysis. *BMJ Open*.

[2] Jiao H., Yan Z., Ma Q. (2018). Influence of Xiaoyaosan on depressive-like behaviors in chronic stress-depressed rats through regulating tryptophan metabolism in hippocampus. *Neuropsychiatric Disease and Treatment*.

[3] Yi L. T., Zhang L., Ding A. W., Xu Q., Zhu Q., Kong L. D. (2009). Orthogonal array design for antidepressant compatibility of polysaccharides from banxia-houpu decoction, a traditional Chinese herb prescription in the mouse models of depression. *Archives of Pharmacal Research*.

[4] Zhou X. J., Liu M., Yan J. J., Cao Y., Liu P. J. J. (2012). Antidepressant-like effect of the extracted of Kai Xin San, a traditional Chinese herbal prescription, is explained by modulation of the central monoaminergic neurotransmitter system in mouse. *Journal of Ethnopharmacology*.

[5] Li X., Wu T., Yu Z. (2018). Apocynum venetum leaf extract reverses depressive-like behaviors in chronically stressed rats by inhibiting oxidative stress and apoptosis. *Biomedicine & Pharmacotherapy*.

[6] Engel D. F., de Oliveira J., Lieberknecht V., Rodrigues A. L. S., de Bem A. F., Gabilan N. H. (2018). Duloxetine protects human neuroblastoma cells from oxidative stress-induced cell death through akt/nrf-2/HO-1 pathway. *Neurochemical Research*.

[7] Hu Y., Chen C., Wang Y. (2021). The effects of KaiXinSan on depression and its association with lipid profiles: a randomized, double-blinded, placebo-controlled trial. *Phytomedicine*.

[8] Chen L., Wang X., Zhang Y. (2021). Daidzein alleviates hypothalamic-pituitary-adrenal Axis hyperactivity, ameliorates depression-like behavior, and partly rectifies circulating cytokine imbalance in two rodent models of depression. *Frontiers in Behavioral Neuroscience*.

[9] Li Y., Zhang D., Li L. (2021). Ginsenoside Rg1 ameliorates aging-induced liver fibrosis by inhibiting the NOX4/NLRP3 inflammasome in SAMP8 mice. *Molecular Medicine Reports*.

[10] Xiong J., Yang J., Yan K., Guo J. J. M. (2021). Ginsenoside Rk1 protects human melanocytes from H_2_O_2_‑induced oxidative injury via regulation of the PI3K/AKT/Nrf2/HO‑1 pathway. *Molecular Medicine Reports*.

[11] Shi Q., Chen J., Zhou Q. (2015). Indirect identification of antioxidants in polygalae radix through their reaction with 2, 2-diphenyl-1-picrylhydrazyl and subsequent HPLC-ESI-Q-TOF-MS/MS. *Talanta*.

[12] Yan L., Mahady G., Qian Y. (2020). Wei MJE-bc, eCAM am: acorus tatarinowiiThe essential oil from Acori tatarinowii rhizome (the dried rhizome of Schott) prevents hydrogen peroxide-induced cell injury in PC12 cells: a signaling triggered by CREB/PGC-1 activation. *Evidence-Based Complementary and Alternative Medicine*.

[13] Fang C., Paul C. R., Day C. H. (2021). Poria cocos (fuling) targets TGF*β*/Smad7 associated collagen accumulation and enhances Nrf2-antioxidant mechanism to exert anti-skin aging effects in human dermal fibroblasts. *Environmental Toxicology*.

[14] Ru J., Li P., Wang J. (2014). TCMSP: a database of systems pharmacology for drug discovery from herbal medicines. *Journal of Cheminformatics*.

[15] Xue R., Fang Z., Zhang M., Yi Z., Wen C., Shi T. J. N. (2012). TCMID: traditional Chinese medicine integrative database for herb molecular mechanism analysis. *Nucleic Acids Research*.

[16] Wu Y., Zhang F., Yang K. (2019). SymMap: an integrative database of traditional Chinese medicine enhanced by symptom mapping. *Nucleic Acids Research*.

[17] Piñero J., Ramírez-Anguita J. M., Saüch-Pitarch J. (2020). The DisGeNET knowledge platform for disease genomics: 2019 update. *Nucleic Acids Research*.

[18] UniProt Consortium (2021). UniProt: the universal protein knowledgebase in 2021. *Nucleic Acid Research*.

[19] Kanehisa M., Sato Y., Kawashima M. J. P.P. S. (2022). KEGG mapping tools for uncovering hidden features in biological data. *Protein Science*.

[20] Panossian A. G., Efferth T., Shikov A. N. (2021). Evolution of the adaptogenic concept from traditional use to medical systems: pharmacology of stress- and aging-related diseases. *Medicinal Research Reviews*.

[21] Yin J., Lin R., Wu M. (2021). Strategy for the multi-component characterization and quality evaluation of volatile organic components in kaixin san by correlating the analysis of headspace-gas chromatography-ion mobility spectrometry and headspace-gas chromatography-mass spectrometry. *Rapid Communications in Mass Spectrometry*.

[22] Hu Y., Liu X., Zhang T. (2020). Behavioral and biochemical effects of KXS on postmyocardial infarction depression. *Frontiers in Pharmacology*.

[23] Wang Y., Wang Y., Chen C. (2021). A randomized, placebo-controlled, double-blind study on the effects of szl on patients with mild to moderate depressive disorder with comparison to fluoxetine. *Journal of Ethnopharmacology*.

[24] Gao W., Wang W., Peng Y., Deng Z. J. M. (2019). Antidepressive effects of kaempferol mediated by reduction of oxidative stress, proinflammatory cytokines and up-regulation of AKT/*β*-catenin cascade. *Metabolic Brain Disease*.

[25] Chen L. x., Qi Z., Shao Z. j. (2019). Study on antidepressant activity of pseudo-ginsenoside HQ on depression-like behavior in mice. *Molecules*.

[26] Dong X. Z., Li Z. L., Zheng X. L., Mu L. H., Zhang G. q, Liu P. J. J. (2013). A representative prescription for emotional disease, ding-zhi-xiao-wan restores 5-HT system deficit through interfering the synthesis and transshipment in chronic mild stress-induced depressive rats. *Journal of Ethnopharmacology*.

[27] Zhang S. J., Wang Q., Liang W. X. (2019). Kai xin san ameliorates scopolamine-induced cognitive dysfunction. *Neural Regeneration Research*.

[28] Jiang N., Wang H., Li C. (2021). The antidepressant-like effects of the water extract of panax ginseng and polygala tenuifolia are mediated via the BDNF-TrkB signaling pathway and neurogenesis in the hippocampus. *Journal of Ethnopharmacology*.

[29] Yan L., Wei M., Gong A. G. (2017). A modified Chinese herbal decoction (kai-xin-san) promotes NGF-induced neuronal differentiation in PC12 cells via up-regulating Trk A signaling. *Frontiers in Cell and Developmental Biology*.

[30] Dong X. Z., Wang D. X., Lu Y. P. (2017). Antidepressant effects of kai-xin-san in fluoxetine-resistant depression rats. *Brazilian Journal of Medical and Biological Research*.

[31] Wang N., Jia Y. M., Zhang B. (2017). Neuroprotective mechanism of *kai xin san*: upregulation of hippocampal insulin-degrading enzyme protein expression and acceleration of amyloid-beta degradation. *Neural Regeneration Research*.

[32] Zhu Y., Duan X., Huang F. (2016). Kai-xin-san, a traditional Chinese medicine formula, induces neuronal differentiation of cultured PC12 cells: modulating neurotransmitter regulation enzymes and potentiating NGF inducing neurite outgrowth. *Journal of Ethnopharmacology*.

[33] Guo S., Wang J., Xu H. (2019). Classic prescription, kai-xin-san, ameliorates alzheimer’s disease as an effective multitarget treatment: from neurotransmitter to protein signaling pathway. *Oxidative Medicine and Cellular Longevity*.

[34] Shuster A., Rocha F., Wayszceyka S. (2021). Protective effect of myrcia pubipetala miq. against the alteration s in oxidative stress parameters in an animal model of depression induced by corticosterone. *Brain Resaerch*.

[35] Herbet M., Szumełda I., Piątkowska-Chmiel I., Gawrońska-Grzywacz M., Dudka J. (2021). Beneficial effects of combined administration of fluoxetine and mitochondria-targeted antioxidant at in behavioural and molecular studies in mice model of depression. *Behavioural Brain Research*.

[36] Wu X., Wang J., Song L. (2021). Catalpol weakens depressive-like behavior in mice with streptozotocin-induced hyperglycemia via PI3K/AKT/Nrf2/HO-1 signaling pathway. *Neuroscience*.

[37] Guo Y., Yan S., Gong J., Jin L., Shi B. J. B. (2018). The protective effect of selenium on bovine mammary epithelial cell injury caused by depression of thioredoxin reductase. *Biological Trace Element Research*.

[38] Bharti V., Tan H., Deol J., Wu Z., Wang J. F. (2020). Upregulation of antioxidant thioredoxin by antidepressants fluoxetine and venlafaxine. *Psychopharmacology*.

[39] Rosa J. M., Pazini F. L., Cunha M. P. (2018). Antidepressant effects of creatine on amyloid *β*1–40-treated mice: the role of GSK-3*β*/Nrf2 pathway. *Progress in Neuro-Psychopharmacology and Biological Psychiatry*.

